# Risk Factors of Enterostomy Infection Caused by Bacterial Infection through Mathematical Modelling-Based Information Data Analysis

**DOI:** 10.1155/2021/4634659

**Published:** 2021-10-16

**Authors:** Jing Li, Xiaoyu Liu, Jun Chen

**Affiliations:** Gastrointestinal Surgery, Chongqing University Cancer Hospital, No. 181 Hanyu Road, Shapingba District, Chongqing 400030, China

## Abstract

**Objective:**

The study aimed to explore the risk factors of infections after enterostomy through the information data analysis method based on a mathematical model.

**Methods:**

156 cases of enterostomy patients admitted to the hospital were retrospectively selected as the study subjects and were divided into the infection group (17 cases) and normal group (139 cases) according to whether they were complicated with infections. Then, the factors of infection and related indexes before and after surgery were analyzed, and the data of the whole hospital were estimated by mathematical modelling.

**Results:**

The length of hospital stay in the infection group was 21 ± 11.2 days, which is longer than 10.1 ± 7.1 days in the normal group (*P* < 0.05). The incidence of anastomotic fistula in the infection group was 14%, which is higher than 2% in the normal group. The mortality rate of infection group (44%) was higher than that of normal group (5%). In the infection group, the incidence of single-cavity stoma (69%) was higher than that of double-cavity stoma (31%), the nosocomial infection rate (11%) was significantly higher compared with out of hospital (2%), and there were significant differences (*P* < 0.05).

**Conclusions:**

Patients with malnutrition and hypoproteinemia before enterostomy, the use of gastric tube and ventilator in the treatment, single lumen stomy in the operation, and the occurrence of anastomotic fistula were more likely to have concurrent infections.

## 1. Introduction

Enterostomy is a common surgical treatment for certain gastrointestinal diseases, which can effectively improve the quality of life of patients [1]. The specific operations of this method are to make an artificial wound in the abdomen of the human body and then suture the opening of the digestive tract so that the patient can excrete waste from the human body through this opening [2]. Patients who undergo the enterostomy often need to have their original diseases treated before permanent or temporary enterostomy, which will change the fecal excretion mode [3]. However, the waste discharged from the stoma cannot be controlled and often flows out involuntarily, soaking the abdominal skin around the stoma. Moreover, the excrement contains many bacteria, which often infect the stoma and surrounding tissues to cause complications, so that the quality of life of patients will be affected [4]. According to reports, the number of patients undergoing ostomy in Taiwan has increased by about 100,000 each year and the number of patients with early complications is about 6.3%–53.8% [5].

Among the many complications, the incidence of stoma infection is higher [6]. The common complications of ostomy include wound infections near the stoma, infections caused by sutures, detachment of the stoma mucosa, and complications caused by the patient's own factors. The above complications will have a serious impact on the patient's postoperative physiology and psychology, which also indirectly lead to unsatisfactory postoperative recovery [7]. In addition, the body's immunity will decrease after surgery and the integrity of the skin and mucous membranes will be destroyed, resulting in open wounds, especially the excretion of feces. Worse still, the stoma and surrounding tissues are prone to bacterial infections, and severe cases may even cause systemic acute infections due to local infections [8].

As its name suggests, mathematical modelling is the process to establish a mathematical model based on actual data information to deal with the problems in reality [9]. Specifically, information data are transformed from basic to in-depth and from rough adjustment to high precision so that more meaningful and usable information can be obtained from simple numbers to solve practical problems in life. It is also a process of integrating theory with practice [10, 11]. The establishment of mathematical models is diverse, and it has been extensively used in various industries, such as medicine and education [12, 13].

In this study, mathematical modelling was introduced to analyse the possible risk factors of bacterial infections after enterostomy, and the obtained data information was adopted in medical practice, which is expected to provide a certain theoretical basis for the prevention of complications caused by enterostomy.

## 2. Experimental Methods

### 2.1. Research Objects

156 patients admitted to hospital for acute enterostomy from September 2018 to January 2021 were taken as the research subjects, including 89 male patients and 67 female patients, aged 54–89 years, with an average age of 56 ± 9 years, and they were rolled into the infection group (*n* = 17) and the normal group (*n* = 139) based on whether they had complicated infections. The criteria for infection were the white blood cell (WBC) count greater than 10 × 10^9^/L, neutrophils greater than 80%, or were accompanied by cough, chest tightness, dyspnea, and other symptoms. One patient with 4 or more of the above could be diagnosed. The study had been approved by the ethics committee of hospital, and the patients and their family members understood the content and methods of this study and agreed to sign the corresponding informed consent.

  Inclusion criteria: (1) all patients were between 50 and 90 years old, (2) patients and their families signed the informed consent, (3) patients were conscious during the study, and (4) the general clinical data of the patients were complete.
  Exclusion criteria: (1) patients with heart, liver, and kidney dysfunction and (2) women in pregnancy.

### 2.2. Research Methods

In this study, a retrospective analysis was conducted on the postoperative development of the enterostomy in hospital, and the general data and clinical treatment data of the research subjects were sorted out for comparative analysis. Besides, the conditions of all patients in the hospital were explored on the basis of mathematical modelling.

### 2.3. Observation Indicators

The etiology of enterostomy in patients was analyzed, and the probability of infections in patients with different variables was compared. Different variables included factors such as stoma intestinal segment, anastomosis method, age, stoma-reduction interval, surgical time, postoperative hospital stay, postoperative anastomotic fistula, postoperative intestinal obstruction, and other factors.

The general information status of patients was compared for statistical significance, including gender, age, and etiology of the stoma.

According to the infection of enterostomy, the patients were divided into groups and compared for hypoproteinemia, the use history of gastric tube and ventilator, the postoperative malnutrition, and the stoma method. Besides, the mortality rate of the infected patients was also counted.

### 2.4. Analysis Method Based on Mathematical Modelling

The mathematical modelling was constructed based on randomly selected patients undergoing enterostomy, so as to estimate the conditions of all patients in the entire hospital.

In order to estimate the number of enterostomy patients with concurrent infection in the whole hospital, the number of enterostomy patients with concurrent infection in the hospital was set as *f*(*x*), the number of randomly selected patients who underwent enterostomy was set as *y*, the number of infected cases was set as *x*, and the total number of patients undergoing enterostomy in the whole hospital was set as *f*(*y*). Then, equation (1) could be obtained:

(1) $$\begin{array}{c} f\left(x\right)=f\left(y\right)\times \frac{x}{y}. \end{array}$$

Thus, the number of patients without concurrent infection in the whole hospital *f*(*x*′) could be expressed in equations (2) and (3):

(2) $$\begin{array}{c} f\left(x^{\prime }\right)=f\left(y\right)-f\left(x\right), \end{array}$$

(3) $$\begin{array}{c} f\left(x^{\prime }\right)=f\left(y\right)-\left(f\left(y\right)\times \frac{x}{y}\right). \end{array}$$

The number of patients with concurrent infections caused by this factor in the whole hospital could be set as *M* to understand the proportion of concurrent infections after surgery caused by different factors in the whole hospital, and the number of cases with this cause in the randomly selected patients was set as *M*′. The calculation is shown in equations (4) and (5):

(4) $$\begin{array}{c} \frac{M}{f\left(x\right)}=\frac{M{}^{\prime }}{x}, \end{array}$$

(5) $$\begin{array}{c} M=\frac{M{}^{\prime }}{x}\times \left(f\left(y\right)\times \frac{x}{y}\right). \end{array}$$

Among them, the number of randomly selected patients who underwent enterostomy (*y*), the number of the infected patients (*x*), and the total number of patients who received enterostomy in the hospital (*f*(*y*)) were all the known quantity.

### 2.5. Statistical Methods

SPSS19.0 software was used for statistical analysis of the data, and the measurement data were expressed as mean ± standard deviation. One-way analysis was adopted for analysis. The Wilcoxon rank-sum test or *t*-test was used for measurement data, and count data were detected by the chi-square test or Fisher's exact test. In addition, *P* < 0.05 meant that the difference was statistically substantial.

## 3. Results

### 3.1. Comparison on the Incidence of Infection Caused by Different Factors

Table 1 shows the relationship between the occurrence of incision infection and gender and age. In the infection group, there were 11 males and 6 females. In the normal group, there were 78 males and 61 females. The average age of infected patients was 54 ± 7 years, and the average age of the uninfected was 57 ± 6 years, with no statistical significance (*P* > 0.05).  Table 2 shows the relationship of the ostomy-reduction interval, operation time, and postoperative hospital stay with the incidence of infection. The length of stay in the infection group was 21 ± 11.2 days, which is longer than 10.1 ± 7.1 days in the normal group (*P* < 0.05).  Figure 1 shows different intestinal sites for ostomy. It was found that there was no significant relationship between the intestinal site of ostomy and the incidence of infection (*P* > 0.05).  Figure 2 shows the relationship between anastomotic fistula and the incision infection. The analysis showed that the incidence of anastomotic fistula in the infection group (14%) was higher than that in the normal group (2%) (*P* < 0.05). It can be concluded that there is a certain relationship between the postoperative hospital stay and postoperative anastomotic fistula with the incidence of infection.

There were a total of 350 patients undergoing enterostomy between September 2020 and March 2021 in this hospital. The etiology was then statistically analyzed, and the etiology distribution of patients with enterostomy in the whole hospital was estimated using the analytical method based on mathematical modelling, as shown in Figure 3. Among them, 122 cases were caused by colorectal cancer and obstruction, accounting for 34.8% of the number of enterostomy cases; 88 cases with colorectal trauma accounted for 25%; 35 cases with anastomotic fistula after colorectal cancer surgery accounted for 10%; 21 cases with colorectal perforation accounted for 6%; 17 cases suffered from intestinal obstruction (5%); 21 cases (6%) suffered from surgery/colonoscopy side injury; 12 patients had intestinal strangulation due to volvulus, accounting for 3.4%; and 13 cases had congenital megacolon, accounting for 3.7%. In addition, there were 21 patients with other etiologies, accounting for 6%.

### 3.2. Age and Gender Distribution of the Two Groups of Patients

After grouping, the general data of patients from the two groups were compared and evaluated (Table 3). It was found that there were no significant differences between the basic information of the two groups of patients (*P* > 0.05).

### 3.3. Comparison on the Typical Stoma Status between the Normal Group and the Infection Group

#### 3.3.1. Comparison on the Dermatitis around the Stoma

Figure 4(a) indicates that the patient's intestinal stoma was in a good state. There was no atrophy of the stoma, and there was no separation between the stoma and the surrounding skin tissue. Besides, the skin tissue around the stoma showed a normal state, without obvious redness, depression, and other symptoms.  Figure 4(b) presents the stoma with poor healing after complicated infection. It was found that the stoma was in a shrinking state, and it was separated from the surrounding skin tissue. Moreover, the skin around the stoma had obvious redness, swelling, and depression symptoms.

#### 3.3.2. Comparison on the Separation of the Stoma Mucosa

The intestinal stoma of one patient was in a good state after the surgery (Figure 5(a)), showing that there was no separation of the skin and mucosal tissue around the stoma. In Figure 5(b), the separation of the intestinal stoma and mucosal tissue could be clearly observed, and the surrounding skin had slight redness. Furthermore, it mainly occurred in the early stage after the surgery.

### 3.4. Comparison on Relevant Indicators of Patients from the Two Groups

The two groups were compared for relevant indexes, such as the history of gastric tube application, history of ventilator application, malnutrition, and hypoproteinemia. It was found that the proportion of these cases in the normal group was lower than that of the infection group. The mortality rate of the infection group was as high as 44%, while the mortality rate of patients in the normal group was only 5%, with obvious statistical significance (*P* < 0.05), as shown in Figure 6. In terms of the stoma methods, 69% of patients in the infection group had single-cavity stoma and 31% of patients had double-cavity stoma. Besides, 40% of patients had single-cavity stoma and 60% had double-cavity stoma in the normal group, suggesting that the single-cavity stoma would increase the chance of infection (Figure 7).

### 3.5. Comparison on the Conditions of Infection between In-Hospital and Out-of-Hospital Patients

Based on the results in Section 3.1, the infection rate of the hospitalized patients and out-of-hospital patients was further compared. It was found that the incidence of concurrent infections in hospitalized patients (11%) was higher than that of discharged patients at home (5%), with significant statistical differences (*P* < 0.05), as shown in Figure 8.

## 4. Discussion

According to statistics, postoperative infection types mainly includes infections at the surgical site, lung, and urinary system, and about 3%–44% of colorectal cancer patients develop surgical site infection after surgery [14]. Moreover, postoperative infection seriously affects the prognosis of patients after surgical treatment. The study showed that the number of patients with colorectal cancer complicated with obstruction was the largest, accounting for 34.8% of the total number of colorectal cancer cases, indicating that most patients with colorectal cancer required enterostomy, but there were differences between patients in different countries. Carlsson et al. [15] concluded that colonic diverticulitis was the second cause of colorectostomy in that region, which was different from colorectal trauma ranking second in this study. Roque-castellano et al. [16] found that most of the patients requiring this operation suffered from nontumor diseases. The study results of Desay et al. [17] showed that the probability of tumor patients requiring ostomy and reductive surgery was only 13%, and the effective rate of this method reached 70%. The above study results clearly show the individual differences between patients in China and those in Western countries.

Some studies have suggested that old age seems to be a risk factor [18]. However, the results of this study showed that the incidence of postoperative complications after enterostomy was not significantly related to age (*P* > 0.05). It was found that postoperative coinfection was significantly related to postoperative hospital stay and whether postoperative anastomotic fistula occurred (*P* < 0.05). A longer postoperative hospital stay will lead to a higher infection rate. Based on this, the infection rate of hospitalized patients and out-of-hospital patients was analyzed, and it was found that the nosocomial infection rate was higher compared with the out of hospital. Hospitalized patients have to have tests for postoperative efficacy and physical indicators of detection, which to a certain extent can reduce the body resistance and immune suppression and increase the vulnerability to infection. Moreover, there are so many people in hospital, including the patients, ward staff, the patient's family and friends, and health care workers, and they can all be regarded as carriers of the bacteria [19]. At home, although the nursing is not so professional as that in hospital, but there are few people around, so the probability of infection is lower in a certain extent.

In this study, the patients in the hospital were sampled randomly. The mathematical model established in Section 2.4 was employed to calculate, and then, the concurrent infections of all the patients in the hospital could be estimated. If a nationwide sampling survey is conducted, the mathematical modelling algorithm can also be adopted to estimate the postoperative infections after enterostomy in Taiwan. Mathematical modelling is to solve and optimize actual problems by calculations in the computer. After the data and information are processed, variables are introduced through abstract hypotheses and actual problems are expressed through mathematical theoretical knowledge to deal with actual problems. Wang et al. [20] applied mathematical modelling to analyse the data of traditional Chinese medicine and concluded that the modelling had good data analysis capabilities. Thus, it had certain guiding significance for the synthesis of Chinese patent medicines.

## 5. Conclusion

In the study, 156 cases of enterostomy patients were retrospectively selected as the study subjects and were divided into the infection group (17 cases) and normal group (139 cases) according to whether they were complicated with infections. The factors of infection and related indexes before and after surgery were analyzed, and the data of the whole hospital were estimated by mathematical modelling. In conclusion, patients with malnutrition and hypoproteinemia before enterostomy, the use of gastric tube and ventilator in the treatment, single lumen ostomy in the operation, and the occurrence of anastomotic fistula were more likely to have concurrent infections. However, some limitations in the study should be noted. The sample size is small, which will reduce the power of the study. In the follow-up, an expanded sample size is necessary to strengthen the findings of the study. It is hoped that this study can provide a reasonable theoretical basis for the prevention and treatment of postoperative infection after enterostomy to reduce the postoperative pain of patients and improve the quality of life of patients to a certain extent.

## Figures and Tables

**Figure 1:** Comparison on infection rates of different stoma intestinal segments (*Note.* A: transverse colon; B: ascending colon; C: sigmoid colon).

**Figure 2:** Data results of the anastomotic method, the occurrence of anastomotic fistula, and intestinal obstruction after infection (*Note.* A′: manual suture; B′: instrument anastomosis; C′: anastomotic fistula; D′: intestinal obstruction).

**Figure 3:** Prediction of the distribution of causes of enterostomy in the hospital based on data analysis of mathematical modelling.

**Figure 4:** Comparison between a normal stoma and a stoma with infectious dermatitis. (a) Normal stoma, female, 56 years old. (b) Infectious dermatitis, female, 54 years old.

**Figure 5:** Comparison on mucosal separation between normal stoma and stove mouth. (a) Normal stoma, male, 58 years old. (b) Mucosal separation, male, 57 years old.

**Figure 6:** Comparison on relevant indicators between the two groups of patients (*Note*. W: history of gastric tube application; H: history of ventilator application; Y: preoperative malnutrition; L: hypoproteinemia; S: mortality rate).

**Figure 7:** Comparison on the relationship between two groups of ostomy methods and concurrent infections.

**Figure 8:** Comparison on the conditions of hospital infection and out-of-hospital infection.

**Table 1:** The relationship of the incidence of incision infection with gender and age.

	Male	Female	Age (years)
The total number of cases	89	67	56 ± 9
The number of infected cases	11	6	54 ± 7
The number of noninfected cases	78	61	57 ± 6

**Table 2:** The relationship of the stoma-reduction interval, the surgical time, and the number of days of hospitalization after surgery with the incidence of infection.

	Stoma-reduction interval (M)	Surgical time (min)	Number of days in hospital after surgery (D)
Total average time	7.9 ± 17.9	166.2 ± 80.5	13.2 ± 6.9
Time of infection	15.5 ± 43.9	140.9 ± 56.8	21 ± 11.2
Time of noninfection	7.1 ± 10.9	169.1 ± 83.0	10.1 ± 7.1

**Table 3:** Comparison on general clinical data of patients from the two groups.

	The number of males	The number of females	Age (years)
Infection group	11	6	54 ± 7
Normal group	78	61	57 ± 6

## Data Availability

The data used to support the findings of this study are available from the corresponding author upon request.
